# Aberrantly expressed long non‐coding RNAs in air pollution‐induced congenital defects

**DOI:** 10.1111/jcmm.14645

**Published:** 2019-09-26

**Authors:** Zheng Li, Jianqing Ma, Xingye Li, Matthew T. V. Chan, William K. K. Wu, Zhanyong Wu, Jianxiong Shen

**Affiliations:** ^1^ Department of Orthopaedic Surgery Peking Union Medical College Hospital Chinese Academy of Medical Sciences and Peking Union Medical College Beijing China; ^2^ Department of Orthopedic Surgery The General Hospital of Xingtai Mining Industry Bloc. Orthopaedic Hospital of Xingtai Xingtai China; ^3^ Department of Orthopedic Surgery Beijing Jishuitan Hospital Fourth Clinical College of Peking University Jishuitan Orthopaedic College of Tsinghua University Beijing China; ^4^ Department of Anaesthesia and Intensive Care The Chinese University of Hong Kong Hong Kong China; ^5^ State Key Laboratory of Digestive Diseases Li Ka Shing Institute of Health Sciences The Chinese University of Hong Kong Hong Kong China

**Keywords:** air pollution, congenital spinal malformation, lncRNAs, long non‐coding RNAs

## Abstract

Air pollution has been a serious public health issue over the past few decades particularly in developing countries. Air pollution exposure during pregnancy poses potential threat to offspring as the deleterious substances might pass through placenta to alter foetal development. A growing number of studies have demonstrated that long non‐coding RNAs (lncRNAs) participate in the development of many diseases, including congenital defects. Here, we used RNA sequencing to identify differentially expressed lncRNAs in air pollution‐exposed rat embryos compared with control group. Our data suggested that 554 lncRNAs (216 up‐regulated and 338 down‐regulated) were significantly differentially expressed in the air pollution‐exposed embryos. Moreover, potential cellular functions of these deregulated lncRNAs were predicted via KEGG signal pathway/GO enrichment analyses, which suggested the possible involvements of neurological process, sensory perception of smell and the G‐protein signalling pathway. Furthermore, potential functional network of deregulated lncRNAs and their correlated mRNAs in the development of congenital spinal abnormality was established. Our data suggested that lncRNAs may play a vital role in the pathophysiology of air pollution‐exposed congenital spinal malformation.

## 1 INTRODUCTION

Air pollution has been a serious public health problem over the past decades all over the world.^1^, ^2^, ^3^, ^4^ Previous studies indicated that at least half of the population lived in areas which did not satisfy the World Health Organization (WHO) guidelines—24‐hours mean of 50 μg/m^3^ for PM_10_ (particulate matter <10 μm) and 24‐hours mean of 25 μg/m^3^ for PM_2.5_ (particulate matter <2.5 μm).^5^ Pollutants of air pollution also include gaseous substances, namely ozone, nitrogen oxides and sulphur dioxide.^4^, ^6^, ^7^, ^8^ In this connection, several groups of investigators have reported that there is a strong link between adverse health outcomes including mortality and hospitalization and exposure to air pollution.^9^, ^10^, ^11^ Air pollution exposure during pregnancy is a potential health threat to the unborn child as the pollutants might pass through placenta and affect the developing foetus.^12^, ^13^ Previous studies suggested that exposure to air pollution during pregnancy was linked to behavioural and neuroanatomical abnormalities in the offspring, including impaired intellectual ability, reduction of brain white matter and increased risk of attention deficit/hyperactivity disorder.^1^, ^14^, ^15^ It has also been reported that tobacco is a risk factor for congenital spinal deformities.^16^ However, the molecular events underlying air pollution‐associated congenital defects are still unclear.

Long non‐coding RNAs (lncRNAs) are a group of non‐coding RNAs with >200 nucleotides in length.^17^, ^18^, ^19^ Accumulating evidence suggested that lncRNAs are deregulated in most, if not all, types of human diseases, including tumours, cardiovascular diseases, autoimmune diseases and congenital abnormalities.^20^, ^21^, ^22^, ^23^, ^24^ Mechanistically, lncRNAs modulate gene expression at transcriptional and post‐transcriptional levels and participate in the regulation of a plethora of molecular, cellular and tissue processes, including DNA synthesis, chromatin modification, cell proliferation, apoptosis, differentiation and organ development.^25^, ^26^, ^27^, ^28^ Emerging evidence also suggested that lncRNAs could participate in the pathogenesis of orthopaedic diseases, such as intervertebral disc degeneration, osteoporosis, osteosarcoma and osteoarthritis.^29^, ^30^, ^31^, ^32^, ^33^ To date, the expression, function and the underlying mechanisms of lncRNAs in air pollution‐associated congenital defects are still unknown.

Our group has previously reported on a microRNA signature of air pollution exposure‐induced congenital defects. Herein, using the same platform, we sought to identify deregulated lncRNAs in air pollution‐exposed rat embryos. Our data suggested that 554 lncRNAs (216 up‐regulated and 338 down‐regulated) were significantly differentially expressed in the air pollution‐exposed embryos. Moreover, potential cellular functions of these deregulated lncRNAs were elucidated via KEGG signal pathway/GO enrichment analyses.

## 2 MATERIALS AND METHODS

### 2.1 Animals

Twenty male (Wistar, 20 weeks) and 20 virgin female (Wistar, 20 weeks) rats were purchased from Biotechnology Co. (SPF). These rats were cultured in animal facilities at 22‐24°C under the 12‐hours dark/light cycle. Pregnant rats were divided into the control group (n = 10) and the air pollution‐exposed group (n = 10). The control rats were maintained in an environment of PM_2.5_ < 50 μg/m^3^ with the air purified by an air cleaner while the air pollution‐exposed group was kept in an environment of PM2.5 > 200 μg/m^3^. All of our procedures were approved with the Ethics Committee of Peking Union Medical College Hospital and The General Hospital of Xingtai Mining Industry Bloc (No. ZCKT‐0015).

### 2.2 Sample harvesting

We defined the first day of vaginal plug as GD0 (gestation day). Three embryos from the control group and five embryos from the air pollution‐exposed group were harvested for RNA sequencing.

### 2.3 RNA isolation and sequencing

Total RNA was collected from embryos with TRIzol (Invitrogen) according to the instruction of the manufacturer. The Multiplex RNA centre of Illumina (Illumina, NEB) was utilized to create a sequencing centre, which was then sequenced via 50 nt single‐end on the BGISEQ‐500. LncRNA sequencing was carried out in accordance with a protocol provided by the manufacturer and previous references.^34^, ^35^ Deregulated lncRNAs were defined by the Cuffdiff algorithm using the default parameters. Differentially expressed lncRNAs with *P* < .05 and fold change >2 were subject to further analyses.

### 2.4 KEGG pathway and Gene Ontology analyses

KEGG (Kyoto Encyclopedia of Genes and Genomes) and GO (Gene Ontology) pathway analyses were carried to analyse the functions of the deregulated lncRNAs. Kyoto Encyclopedia of Genes and Genomes signal pathway assay (http://www.genome.jp/kegg/) was used to identify significant signalling pathways. Gene Ontology method was used to identify gene modulator network of lncRNAs of interest in terms of cellular component, biological processes and molecular functions (http://www.geneontology.org).

### 2.5 LncRNAs‐mRNA network reconstruction

To predict the potential functional network of deregulated lncRNAs and their correlated mRNAs in the development of congenital defects, the lncRNA‐mRNA network was established using starBase (http://starbase.sysu.edu.cn/index.php). The lncRNA‐mRNA network was then visualized using Cytoscape.

### 2.6 Statistical analysis

Results were shown as mean ± SD (standard deviation). Student's *t* test was carried out to detect the significant difference. *P* < .05 was considered as statistically significant.

## 3 RESULTS

### 3.1 Dysregulated lncRNAs in air pollution‐exposed embryos

LncRNAs differentially expressed in embryos from the air pollution‐exposed group on GD9 were profiled by lncRNA sequencing. Results showed that 554 lncRNAs were significantly deregulated in embryos with air pollution‐exposed group as compared with the control group, among which 216 and 338 lncRNAs were up‐regulated and down‐regulated, respectively. Deregulated lncRNAs between two groups were visualized with a heatmap (Figure 1A) and the volcano plot (Figure 1B).

**Figure 1:** Differentially expressed lncRNAs in air pollution‐exposed embryos. A, A heatmap representation of all differentially abundant lncRNAs is shown. B, Volcano plots of differentially abundant lncRNAs in air pollution‐exposed embryos. A total of 554 lncRNAs were significantly deregulated in embryos with air pollution‐exposed group as compared with the control group, among which 216 and 338 lncRNAs were up‐regulated and down‐regulated, respectively

### 3.2 KEGG and GO pathway enrichment analyses of deregulated lncRNAs

To study the molecular mechanism via which deregulated lncRNAs take part in the development of congenital defects induced by air pollution, significantly deregulated lncRNAs were chosen to infer the potential molecular functions of their correlated mRNAs (correlation coefficient > .95) using GO and KEGG signalling pathway analyses. The GO is a classification method of gene function with directed acyclic graph (DAG) as an illustration of GO data (Figure 2). The DAG of lncRNA‐regulated biological processes (BP) was found to include the modulation of neurological system process, sensory perception of smell and G‐protein signalling pathway (Figure 3). The DAGs of cellular components (CC) and molecular functions (MF) were shown in Figure 4 and Figure 5, respectively. For KEGG analysis, significantly enriched signalling pathways were sulphur metabolism, ribosome and glycolysis (Figure 6).

**Figure 2:** Functional predictions of differentially abundant lncRNAs in air pollution‐exposed group versus control group by GO (Gene Ontology) assay. The GO is a classification method of gene function with directed acyclic graph (DAG) as an illustration of GO data

**Figure 3:** A and B, Biological processes were predicted to be altered by mRNAs targeted by differentially abundant lncRNAs in air pollution‐exposed group versus control group. The DAG of lncRNA‐regulated biological processes (BP) was found to include the modulation of neurological system process, sensory perception of smell and G‐protein signalling pathway

**Figure 4:** A and B, Cellular components were predicted to be altered by mRNAs targeted by differentially abundant lncRNAs in air pollution‐exposed group versus control group

**Figure 5:** A and B, Molecular functions were predicted to be altered by mRNAs targeted by differentially abundant lncRNAs in air pollution‐exposed group versus control group

**Figure 6:** Scatterplot of enriched KEGG pathway showing statistics of pathway enrichment in air pollution‐exposed group

#### 3.2.1 Reconstruction of lncRNA‐mRNA networks

To infer the potential network of deregulated lncRNAs and their correlated mRNAs in the development of air pollution‐associated congenital defects, we created gene modulator networks of deregulated lncRNAs and their potential target mRNAs. As shown in the Figure 7, an adjustive lncRNA‐mRNA network of differentially expressed (significantly up‐regulated or down‐regulated) lncRNAs and target mRNAs (*P* ≤ .05; fold change >2.0) in the air pollution‐exposed group compared was established.

**Figure 7:** Regulatory networks of lncRNAs and mRNAs between air pollution‐exposed group and control group. An adjustive lncRNA‐mRNA network of differentially expressed (significantly up‐regulated or down‐regulated) lncRNAs and target mRNAs (*P* ≤ .05; fold change >2.0) in the air pollution‐exposed group compared was established

## 4 DISCUSSION

An increasing number of studies have demonstrated that lncRNAs play a key regulatory roles in diverse cellular activities, including differentiation, proliferation and migration and are differentially expressed in most if not all kinds of diseases, including autoimmune, neoplastic, neurodegenerative and orthopaedic diseases.^20^, ^26^, ^36^, ^37^ In this study, we employed RNA sequencing to identify lncRNAs deregulated by exposure to air pollution in rat embryos. Our data suggested that air pollution induced a pervasive deregulation of lncRNAs (216 up‐regulated and 338 down‐regulated). Further bioinformatic analyses suggested that these differentially expressed lncRNAs might regulate neurological system process, sensory perception of smell and G‐protein signalling pathway through interacting with their target mRNAs. In this regard, the lncRNA‐mRNA network was reconstructed. Our data suggested that lncRNA deregulation might take part in the pathogenesis of air pollution‐associated congenital defects.

Previous studies found that lncRNAs may be involved in the development and progression procedure of diseases which are associated with air pollution.^38^, ^39^ For instance, Wei and colleagues found that the lncRNA CAR10 (CAR intergenic 10) was overexpressed in patients with lung cancer from Xuanwei, which has the highest incidence of lung cancer in China due to air pollution.^39^ Lin et al 40 reported that the lncRNA LCPAT1 (lung cancer progression‐association transcript 1) was found to be overexpressed in lung cancer cells after exposure to PM_2.5_ and cigarette smoke extract while inhibition of LCPAT1 expression decreased the pro‐tumorigenic effects of PM_2.5_ and cigarette smoke extract on these cancer cells. He et al 41 also investigated the correlation of lncRNA H19 methylation and DMR methylation together with birth length and weight. Their data showed that prenatal NO_2_ exposure was correlated with increased H19 methylation, whereas PM_10_ exposure and SO_2_ exposure were correlated with reduced H19 DMR and H19 methylation, respectively. Herein, we utilized lncRNA sequencing to analyse lncRNA expression in the embryos on GD9 from control group and air pollution‐exposed group. We selected the GD9 embryos to perform lncRNA sequencing owing to the timing of somitogenesis gradation in rats.^35^ However, it is difficult to detect the congenital defects at this stage. Our study identified 554 lncRNAs differentially expressed in air pollution‐exposed embryos compared with control embryos. These results provided a starting point for research into the possible roles of lncRNAs in pathogenesis of air pollution‐induced congenital defects.

Gene Ontology analysis is an effective bioinformatic technique, which explains the instruction of genes and their specialities pass via species.^42^ Gene Ontology annotations and GO terms were merit prognosis for function and trend of these genes. Kyoto Encyclopedia of Genes and Genomes signal pathway is another effective tool that can give power information for function of genes and was largely used for bioinformatic analysis.^43^, ^44^ Thus, we determined the lncRNA‐dependent gene functions and the association of correlated signalling pathways in pathogenesis of air pollution‐induced congenital malformation using these two methods. Our results demonstrated the possible involvements of neurological system process, sensory perception of smell and G‐protein signalling pathway. Nevertheless, the molecular function and mechanisms of differentially expressed lncRNAs as inferred by the KEGG and GO analyses should be interpreted with caution and validated by functional studies in the future.

In summary, our study suggested that *in utero* exposure to air pollution resulted in pervasive lncRNA deregulation in rat embryos. This lncRNA data set together with the inferred biological functions and lncRNA‐mRNA networks could provide a glimpse into the role of lncRNAs in the development of congenital deformity caused by air pollution.

## CONFLICT OF INTEREST

There is no conflict of interest statement.

## AUTHOR CONTRIBUTION

Zheng Li, Jianqing Ma, Xingye Li, Matthew TV Chan, William KK Wu, Zhanyong Wu and Jianxiong Shen Performed the trials. Zheng Li analysed the data. Zhanyong Wu and Jianxiong Shen contributed reagents. Zheng Li wrote manuscript, and Matthew TV Chan and William KK Wu revised manuscript.
